# Hematocolpos: An Unusual Cause of Right Iliac Fossa Pain

This article has been retracted.

**DOI:** 10.7759/cureus.18835

**Published:** 2021-10-17

**Authors:** Alya A Khashoggi, Nouf A Hakami, Majdoleen A Alghamdi, Hussam Y Ayed, Ali D Alqarni, Talal J Alshahrani, Abdulaziz M Alshamrani, Abdallah S Alayyaf, Raghad A Almansour, Sharouq A Alolyan, Afrah A Alotaibi, Sarah K Alabdulltif, Eman A Obaidi, Hatim A Akkasi, Malak Alshammari

**Affiliations:** 1 College of Medicine, King Saud Bin Abdulaziz University for Health Sciences, Riyadh, SAU; 2 College of Medicine, Jazan University, Jizan, SAU; 3 College of Medicine, King Khalid University, Abha, SAU; 4 College of Medicine, Ibn Sina National College for Medical Studies, Jeddah, SAU; 5 College of Medicine, Prince Sattam Bin Abdulaziz University, Al-Kharj, SAU; 6 College of Medicine, Imam Mohammad Ibn Saud Islamic University, Riyadh, SAU; 7 College of Medicine, Qassim University, Qassim, SAU; 8 College of Medicine, Northern Border University, Arar, SAU; 9 College of Medicine, Taibah University, Medina, SAU; 10 College of Medicine, Majmaah University, Al Majmaah, SAU; 11 College of Medicine, Imam Abdulrahman Bin Faisal University, Dammam, SAU

**Keywords:** case report, hematocolpos, imperforate hymen, abdominal pain, acute appendicitis

## Abstract

Acute appendicitis is the most frequent indication for emergency abdominal surgery in childhood. Despite being a common condition, the diagnosis of acute appendicitis can be challenging. Ultrasound examination remains the imaging tool of choice for the diagnosis of acute appendicitis. We report the case of a nine-year-old girl who presented with acute abdominal pain in the right lower quadrant accompanied by nausea and vomiting. Physical examination revealed right iliac fossa rebound tenderness. Ultrasound examination showed a dilated blind-ended structure in the right iliac fossa conferring the diagnosis of acute appendicitis. The patient underwent a CT scan which made the diagnosis of imperforate hymen with hematocolpos. The patient underwent hymenotomy and her symptoms showed complete resolution. Imperforate hymen with hematocolpos is a rare congenital genital tract anomaly. The case highlights the importance of appropriate genital examination in pediatric patients. In the present case, the patient might have undergone an unnecessary abdominal surgery if the correct diagnosis was not established.

## Introduction

Acute appendicitis is the most frequent indication for emergency abdominal surgery in childhood [1]. Accurate early diagnosis is crucial to prevent the complication of acute appendicitis, such as perforation and abscess formation. Despite being a common condition, the diagnosis of acute appendicitis can be challenging. It usually presents with non-specific gastrointestinal symptoms. Since the history and physical examination have low sensitivity and specificity, imaging has a crucial role in making a prompt and accurate diagnosis. Ultrasound examination remains the imaging tool of choice for the diagnosis of acute appendicitis in children considering its non-invasive nature and carries no ionization radiation [2]. However, the ultrasound has some limitations, importantly it is an operator-dependent examination. Hence, CT had a superior diagnostic performance than ultrasound in diagnosing appendicitis [3]. Here, we describe the case of a young girl who was thought to have acute appendicitis based on the clinical and sonographic findings. However, CT scan revealed the diagnosis of imperforate hymen presenting with a clinical picture of acute appendicitis.

## Case presentation

We present the case of a nine-year-old girl who was brought to the emergency department (ED) with a complaint of abdominal pain for two days duration. The pain was started in the periumbilical region then shifted to the right iliac fossa. Her pain started gradually and has increased in severity. She described it as a constant pain that was not relieved by oral simple analgesic medications. The pain was exacerbated by movement and was not related to posture or meals. She scored the pain as 7 out of 10 in severity. The pain was associated with nausea and few episodes of vomiting that had food content with no blood. One day after the onset of pain, the patient developed a low-grade fever that measured 37.9℃ and was relieved by antipyretics. The parents reported that her daughter had decreased appetite and activity since the onset of pain. However, there was no change in her urinary or bowel habits.

The past medical history of the patient was significant for poorly controlled asthma. She required three admissions in the past year due to asthma exacerbation. She was on an inhaled corticosteroid therapy and short-acting inhaled salbutamol. The patient did not have any surgical history. She attained normal growth and development milestones at an appropriate normal age. The gynecologic history was not obtained from the patient. The patient was a primary school student. There was no history of diseases running in their family and the parents were not consanguineous.

Upon examination, the patient appeared tired and sick. She was not in respiratory distress. She did not appear pale, jaundice, or cyanosed. Her vital signs were a pulse rate of 100 bpm, blood pressure of 98/65 mmHg, respiratory rate of 13 bpm, and temperature of 37.2℃. Abdominal examination revealed a soft and lax abdomen. There was a localized tenderness in the right iliac fossa with rebound tenderness. Cardiorespiratory and neurological examination findings were normal. Initial laboratory findings were suggestive of an active inflammatory process with elevated leukocyte count and inflammatory markers (Table 1). In light of the clinical and laboratory findings, the initial diagnosis was acute appendicitis.

**Table 1:** Summary of the results of laboratory findings.

Laboratory investigation	Unit	Result	Reference range
Hemoglobin	g/dL	13.2	13.0–18.0
White blood cell	1000/mL	13.5	4.0–11.0
Platelet	1000/mL	375	140–450
Erythrocyte sedimentation rate	mm/hr.	26	0–20
C-reactive protein	mg/dL	13.5	0.3–10.0
Total bilirubin	mg/dL	0.7	0.2–1.2
Albumin	g/dL	4.2	3.4–5.0
Alkaline phosphatase	U/L	52	46–116
Gamma-glutamyltransferase	U/L	44	15–85
Alanine transferase	U/L	34	14–63
Aspartate transferase	U/L	28	15–37
Blood urea nitrogen	mg/dL	8	7–18
Creatinine	mg/dL	0.7	0.7–1.3
Sodium	mEq/L	136	136–145
Potassium	mEq/L	3.8	3.5–5.1
Chloride	mEq/L	101	98–107

The patient underwent an abdominal ultrasound examination. It revealed a dilated blind-ended structure in the right iliac fossa with a distended bladder (Figure 1). Such findings were in keeping with the diagnosis of acute appendicitis. The patient underwent a CT scan of the abdomen which revealed marked distension of the vagina with fluid and was displacing the urinary bladder anteriorly. These unexpected findings were in keeping with the diagnosis of hematocolpos and imperforate hymen (Figure 2). The patient was then prepared for hymenotomy under general anesthesia. The procedure resulted in a complete resolution of the patient’s symptoms. She was discharged on the third postoperative day. In the follow-up visits, the patient had no active issues.

**Figure 1:** Ultrasound images. Abdominal ultrasound images demonstrating a distended fluid-filled structure in the suprapubic region (A) and a dilated blind-ended tubular structure in the right iliac fossa (B). These were incorrectly interpreted as the urinary bladder and the appendix, respectively. However, these structures are the blood-filled uterus and dilated right fallopian tube.

**Figure 2:** CT images. Selected CT images in the sagittal (A) and the axial (B) plane demonstrating a markedly dilated uterus (long arrow) displacing the bladder (short arrow) anteriorly.

## Discussion

We presented the case of a young girl with imperforate hymen with a clinical and sonographic picture mimicking acute appendicitis. Imperforate hymen is a rare genital tract anomaly with an incidence of one in 2000 girls [4]. It results from the failure of canalization of the vaginal plate during fetal development. Imperforate hymen usually presents with amenorrhea and cyclic pelvic pain. In the present case, the presentation was very unusual. As a result of the imperforate hymen, the menstrual blood accumulates in the vagina causing marked distention which could exert the pressure effect on the bladder and the urethra. Up to 50% of patients with hematocolpos usually present with acute urinary retention [5]. The menarche is typically the trigger for the clinical presentation of this condition. However, on extremely rare occasions, an imperforate hymen may present in the neonatal period with mucocolpos [1]. 

While the diagnosis of imperforate hymen sounds straightforward, the diagnosis is often delayed or missed in the clinical practice because physicians do not usually obtain a detailed gynecological history of performing gynecological examination routinely [6]. In the present case, neither the gynecological history nor the appropriate physical examination was performed.

Ultrasound examination usually makes the diagnosis. However, in the present case, the radiologists were preoccupied with the initially provided clinical data of acute appendicitis. Hence, the abnormally fluid-filled uterus was incorrectly interpreted as the urinary bladder. Similarly, the abnormally dilated fallopian tube in the right iliac fossa was incorrectly interpreted as the appendix. It is well known that the clinical data provided to the radiologists may cause a distraction and leads to false-positive interpretations [5].

The management of imperforate hymen with hematocolpos is hymenotomy. While this procedure is curative for imperforate hymen, regular follow-up is essential as some patients experience recurrence of symptoms. Some authors advocate performing a virginity-sparing procedure because of cultural and religious aspects [7].

## Conclusions

Imperforate hymen with hematocolpos is a rare congenital genital tract anomaly. Clinicians should keep a high index of suspicion for this condition when they encounter an adolescent pre-menarche girl presenting with abdominal pain. The case highlights the importance of appropriate genital examination in pediatric patients. In the present case, the patient might have undergone an unnecessary abdominal surgery if the correct diagnosis was not established.
